The article "Inflammatory myofibroblastic tumor with RANBP2 and ALK gene rearrangement: a report of two cases and literature review" was published in 2013. Journal: Diagn Pathol.

# Inflammatory myofibroblastic tumor with *RANBP2* and *ALK* gene rearrangement: a report of two cases and literature review

**DOI:** 10.1186/1746-1596-8-147

**Published:** 2013-09-13

**Authors:** Jian Li, Wei-hua Yin, Kengo Takeuchi, Hong Guan, Yu-hua Huang, John KC Chan

**Affiliations:** 1 Department of Pathology, Peking University Shenzhen Hospital, No. 1120, Lianhua North Road, Shenzhen 518000, China; 2 Pathology Project for Molecular Targets of the Cancer Institute, Tokyo 135-8550, Japan; 3 Division of Pathology of the Cancer Institute Hospital, Japanese Foundation for Cancer Research, 3-8-31 Ariake, Koto, Tokyo 135-8550, Japan; 4 Department of Pathology, the Second Shenzhen People’s Hospital, Sungang West Road, Shenzhen 518035, China; 5 Department of Pathology, Queen Elizabeth Hospital, Hong Kong, SAR, China

**Keywords:** Inflammatory myofibroblastic tumor, RANBP2-ALK, Fluorescence in situ hybridization

## Abstract

**Abstract:**

Inflammatory myofibroblastic tumors (IMTs) are categorized as intermediate biologic neoplasms, whereas IMTs with genetic features of ran-binding protein 2 (*RANBP2*) and anaplastic lymphoma kinase (*ALK*) rearrangement (IMT-RAs) are possibly related to a more aggressive clinical course. However, fewer than 10 cases of IMT-RA have been reported to date. Herein, we present 2 new cases of IMT-RA in which both tumors recurred quickly after primary surgery; one patient died 3 months later from the disease, and the other patient has been living with the disease for 12 months. IMT-RAs are characterized by noncohesive epithelioid and rounded tumoral cell morphology, commonly derived from pelvic and peritoneal cavities, and frequently show larger tumor sizes. The relation between the clinicopathologic features and poor prognosis of IMT-RA is discussed.

**Virtual slides:**

The virtual slide(s) for this article can be found here: http://www.diagnosticpathology.diagnomx.eu/vs/3314123381007714

## Background

Inflammatory myofibroblastic tumors (IMTs) are mesenchymal neoplasms of intermediate biologic potential that are derived from myofibroblastic cells and accompanied by rich inflammatory infiltrates [1]. IMTs have a predilection for children and adolescents, and the most common anatomical locations are the abdominopelvic region, lung, and retroperitoneum. IMTs show expression of anaplastic lymphoma kinase (ALK) protein triggered by *ALK* gene (at 2p23) rearrangement, which has been found in 36–60% of IMTs [2]. ALK fusion oncogenes have been identified in a small proportion of IMTs, including *SEC31L1* at 4q21, *ATIC* at 2q35, *CARS* at 11p15, *TPM3* at 1p23, *TMP4* at 19p13, *CLTC* at 17q23, *PPFIBP1* at 12p11, and ran-binding protein 2 (*RANBP2*) at 2q13 [3]. Different fusion partners may lead to distinct subcellular locations of the corresponding chimeric protein, which result in distinct immunostaining patterns when detected by ALK antibody. IMTs with CARS, ATIC, and SEC31L1 fusion are generally associated with smooth cytoplasmic staining, whereas fusion with CLTC, a main structural protein of coated vesicles, displays a granular cytoplasmic pattern [4].

The article "Inflammatory myofibroblastic tumor with RANBP2 and ALK gene rearrangement: a report of two cases and literature review" was published in 2013. Journal: Diagn Pathol.

*RANBP2* fuses with the *ALK* gene through balanced or unbalanced translocation [5]. The *RANBP2* gene encodes a 358-kd nuclear pore protein [6], thus IMTs with *RANBP2-ALK* (IMT-RA) rearrangement display a unique nuclear membrane staining pattern. Most importantly, IMT-RA is possibly associated with a poor prognosis; however, this relation remains inconclusive, as fewer than 10 cases of IMTs with genetically confirmed *RANBP2-ALK* fusion have been reported to date [5,7-11]. Herein, we present 2 new cases of IMT-RA with follow-up information. The relations between the histopathologic features and prognosis of IMT-RAs are discussed further.

### Case presentation

Case 1 was a 19-year-old female who was hospitalized due to paroxysmal abdominal pain combined with nausea and vomiting for 4 days. Ultrasound examination showed a 19 × 17 × 11 cm solid mass in the pelvic cavity and medium amounts of ascitic fluid. Intraoperatively, the tumor was situated in the mesenterium region of the terminal ileum, and had locally invaded into the adjacent ileum wall. Resections of the tumor, affected terminal ileum, and ileocecum were performed. The patient rejected further chemotherapy. Nine weeks after the operation, radiological imaging displayed recurrent intra-abdominal occupations with massive ascites. Concurrently, acute renal insufficiency was identified by laboratory tests. The patient died of the disease after 3 weeks of maintenance treatment.

Case 2 was a 39-year-old male with an initial complaint of laborious urination for more than 2 months and abdominal distention and abdominal pain for 10 days. Computer Tomography (CT) revealed a 15 × 10 × 8 cm occupation in the pelvic cavity (Figure 1). The neoplasm was found in the mesangial region at the junction of sigmoid and rectum during the operation, with invasions of the neighboring sigmoid, the upper portion of the rectum, and left ureter. The tumor and afflicted intestines and left ureter were completely excised. The patient was treated with epirubicin and iphosphamide following the operation. Four months after the first excision, CT showed multiple recurrent masses in the presacral, pararectal, and left iliac vessel regions. The patient then underwent chemoembolization therapy. Follow-up has continued to date, and the patient has lived with the tumor for 12 months.

The article "Inflammatory myofibroblastic tumor with RANBP2 and ALK gene rearrangement: a report of two cases and literature review" was published in 2013. Journal: Diagn Pathol.

**Figure 1:** Computer tomography of Case 2 revealed a heterogeneous-density occupation in the left pelvic cavity.

### Histopathological and genetic findings

The gross and histological features were similar in Case 1 and Case 2. The tumors were solid and gray-yellowish in the cut surface. Focal hemorrhage and a myxomatous appearance were observed. Microscopically, the neoplasm showed a fasciitis-like pattern and the stromal myxoid change was prominent (Figure 2A, B). The tumor cells were generally non-cohesive, and frequently demonstrated ganglion-like morphology of slightly amphophilic cytoplasm, vesicular chromatin, and large nucleoli (Figure 2C). There were also a few binucleate cells sparsely presented in the lesion (Figure 2D). In area of the neoplasm, some tumor cells were tightly packed and arranged in sheets (Figure 2E). The mitotic figures ranged from 1 to 4 per 10 high-power fields. There were abundant admixed polymorphs infiltrates, including neutrophils, eosinophils, and lymphoplasma cells, which were unevenly distributed throughout the lesion. Erythrocyte extravasation was another feature found in both cases. The tumor invaded the adjacent intestinal tissues, involving the adventitia, muscularis propria, and submucosa with a vague nodular pattern (Figure 2F).

**Figure 2:** **Histopathological findings of inflammatory myofibroblastic tumor with *RANBP2 *and *ALK *gene rearrangement. (A)** and **(B)** The neoplastic cells were loosely arrayed and distributed in an abundant myxoid stroma. There were striking neutrophilic inflammatory infiltrates in the lesion, while lymphoplasma cells were only occasionally observed (inserted panel) (**A** and **B**, hematoxylin and eosin [H&E] staining, 200× original magnification; inserted panel, H&E staining, 400× original magnification). **(C)** The tumor cells showed ganglion-like morphology, characterized by an abundant and slightly amphophilic cytoplasm, round nuclei, vesicular chromatin, and large nucleoli (H&E staining, 400× original magnification). **(D)** A few binucleate cells were found in the tumor (H&E staining, 400× original magnification). **(E)** In focal area, the tumor cells were tightly packed around dilated vessels (H&E staining, 100× original magnification). **(F)** The tumor infiltrated the adjacent intestinal wall in a vague nodular pattern (H&E staining, 40× original magnification).

Immunohistochemically, the tumor cells showed distinctive nuclear membrane staining for ALK (Dako; Clone ALK1; Ready-to-use) (Figure 3A) in both cases. Similarly, positive staining for CD30 (Dako; Clone Ber-H2; 1:40 dilution) (Figure 3B), desmin (Dako; Clone D33; 1:100 dilution) (Figure 3C), and SMA (Dako; Clone 1A4; 1:100 dilution) was also observed in some tumor cells in the 2 cases. In both cases, the tumor cells were nonreactive to AE1/AE3 (Dako; Clone AE1 + AE3; 1:200 dilution), cytokeratin 8/18 (Santa Cruz Biotechnology; Clone NCL-5D3; 1:100 dilution), CD117 (Dako; polyclonal; 1:100 dilution), calponin (Santa Cruz Biotechnology; Clone CALP; 1:200 dilution), S100 (Dako; polyclonal; 1:500 dilution), CD21 (Dako; Clone 1 F8; 1:25 dilution), HMB45 (Dako; 1:50 dilution), myogenin (Dako; Clone F5D; 1:50 dilution), and Myf4 (Novocastra; Clone LO26; 1:500 dilution).

The article "Inflammatory myofibroblastic tumor with RANBP2 and ALK gene rearrangement: a report of two cases and literature review" was published in 2013. Journal: Diagn Pathol.

**Figure 3:** **Immunohistochemistry features of inflammatory myofibroblastic tumor.** The tumor cells showed nuclear membranous ALK immunostaining **(A)**, cytomembranous CD30 immunostaining **(B)**, and cytoplasmic desmin immunostaining **(C)** (**A** and **B**, 400× original magnification; **C**, 200× original magnification). **(D)** Interphase fluorescence *in situ* hybridization (FISH) revealed 1 fused signal (arrow) in the tumor nucleus, indicating the presence of *RANBP2-ALK* translocation. One separate orange signal and 1 separate green signal indicated a normal *ALK* and a normal *RANBP2* locus, respectively (1000× original magnification).

Fluorescence *in situ* hybridization (FISH) was performed on 4 μm-thick tissue sections with bacterial artificial chromosome probes for *RANBP2* (RP11-348G16) and *ALK* (RP11-984I21 and RP11-62B19). In both cases, 1 fused signal was observed in the tumor cell nucleus, indicating the presence of *RANBP2* and *ALK* gene rearrangement (Figure 3D) by unbalanced genetic rearrangement mechanism [5].

To pinpoint the fusion location of the *RANBP2* and *ALK* genes, reverse-transcription polymerase chain reaction (RT-PCR) analysis was performed. Total RNA was extracted from 15 μm-thick paraffin sections using the RNeasy® FFPE kit (QIAGEN, Germany), and reverse-transcribed using random hexamer primers. PCR was performed using previously introduced primers [8] for 45 cycles as follows: 94°C for 30 seconds, 60°C for 30 seconds, and 72°C for 30 seconds. An expected 254-bp amplification product was detected in Case 2 (Figure 4A). No PCR product was identified in Case 1, which may be due to RNA degradation in the paraffin-embedded block since positive amplification results (285-bp) of beta-actin as a householding gene were not found either in Case 1 but present in Case 2 (Figure 4B). Direct sequencing of the chimeric cDNA product confirmed that the *RANBP2-ALK* fusion point was composed of exon 18 of *RANBP2* to exon 20 of *ALK* (Figure 4C).

**Figure 4:** **Genetic features of inflammatory myofibroblastic tumor. (A)** Reverse-transcription polymerase chain reaction (RT-PCR) with *RANBP2* and *ALK* primers. Lane T1: no amplification band was observed in Case 1. Lane T2: an expected 254-bp product was present in Case 2. Lane C: tonsil tissue was adopted as a control, and no amplification band was observed. Lane NTC: no template control. **(B)** Detection of house-keeping gene of beta-actin by RT-PCR. An expected 285-bp product was seen in Case 2 (Lane 2) and tonsil tissue (Lane 3). No amplification band was observed in Case 1 (Lane 1) and no-template control (Lane NTC). **(C)** The fusion point of the *RANBP2-ALK* gene as indicated by cDNA sequencing was located between exon 18 of the *RANBP2* gene and exon 20 of the *ALK* gene.

The article "Inflammatory myofibroblastic tumor with RANBP2 and ALK gene rearrangement: a report of two cases and literature review" was published in 2013. Journal: Diagn Pathol.

## Discussion

IMT is regarded as a neoplasm of intermediate biologic potential. Overall, the recurrence rate varies by anatomical sites, from 2% for tumors confined to the lung to 25% for extrapulmonary lesions. Distant metastasis of IMT occurs in less than 5% of cases [12]. According to the literature and the 2 cases presented herein (Table 1), the local recurrence rate of IMT-RA is 88% (7/8) with a metastasis rate of 25% (2/8), both markedly higher than those of conventional IMTs. Furthermore, 2 patients (25%, 2/8) have died from the disease within 6 months after the tumor excision. These data suggest that IMT-RAs are more invasive clinically.

**Table 1:** **Clinical features of 11 cases of inflammatory myofibroblastic tumor with *RANBP2-ALK *gene fusion**

**Case**	**Author**	**Age**	**Sex**	**Anatomic site(s)**	**Size (cm)**	**Treatment**	**Follow-up**
1	Ma [5] (2003)	7 y	Male	Unspecified abdominal mass	NA	SE + CT	Recurred 5 weeks later after first resection. A re-excision was performed. Five months later, the tumor recurred again and was re-excised.
2		7 m	Male	Mesentery and omentum	11	SE	Recurred 8 months later after first resection. A re-excision was performed.
3	Patel [7] (2007)	2 y	Male	Retroperitoneal abdominal mass	10	SE	No evidence of recurrence with 3 years of follow-up.
4	Chen [8] (2008)	34 y	Male	Liver	8	SE	Recurred 5 months later after resection. Died of the disease approximately 2 weeks after discovery of the recurrence.
5	Butrynski [9] (2010)	44 y	Male	Omentum	NA	SE + CT + ALKi	Hepatic, peripancreatic, and perirectal masses recurred 1 year later after resection. Subsequent exploratory laparotomy with maximal debulking was performed.
6	Marino-Enriquez [10] (2011)	41 y	Male	Omentum	26	SE + CT + ALKi	Multifocal local recurrence and liver metastases. Alive with no evidence of disease for 40 months.
7		6 y	Male	Omentum and Mesentery	14	SE	NA
8		39 y	Male	Mesentery of the small bowel	14	SE	NA
9	Kozu [11] (2013)	57 y	Male	Pluera or chest wall	NA	ALKi	NA
10	Present cases (2013)	19 y	Female	Mesentery of the small bowel	19	SE	Recurred 9 weeks later after resection. Died of the disease 3 weeks later after discovery of the recurrence.
11		39 y	Male	Mesentery of the colon	15	SE + CT	Recurred 4 months later after resection. Alive with disease for 12 months.

*SE* surgical excision, *CT* chemotherapy, *ALKi* ALK inhibitor, *NA* data not available.

The article "Inflammatory myofibroblastic tumor with RANBP2 and ALK gene rearrangement: a report of two cases and literature review" was published in 2013. Journal: Diagn Pathol.

The aggressive behavior of IMT-RA might be associated with the following aspects: (1) The location and size of the tumor: Coffin et al. [13] analyzed the clinicopathologic features of IMTs with an invasive course, and found that IMTs that arise in the abdominopelvic site are more likely to recur (with a recurrence rate of 85%). In addition, recurrent and metastatic IMTs were commonly larger in size, with mean diameters of 8.7 and 11 cm, respectively. Of the 11 reported cases of IMT-RAs, 10 occurred in the abdominopelvic area, and only 1 presented in the pleural cavity (no follow-up data were provided in the case). The average size on discovery was 14.6 cm. Thus, the aggressiveness of IMT-RA is possibly related at least in part to its abdominopelvic origination and bigger tumor size. It is worth noting that IMT-RA seemingly prefers to afflict male patients, as the male to female ratio is 10:1.

(2) The histological features of the tumor: The morphology of IMT-RAs is generally uniform and characterized by loosely arrayed, ganglion-like or epithelioid neoplastic cells distributed in a widespread myxoid stroma. In earlier reports, IMTs with the aforementioned features were named round cell transformation [14]. It has been well demonstrated that IMTs with round cell transformation behave aggressively with rapid recurrence and/or death, compared to conventional IMTs in which spindled tumoral cells predominate [14]. Marino-Enriquez [10] proposed to designate this type of IMT as epithelioid inflammatory myofibroblastic sarcoma based on its histological and malignant biological characteristics. Therefore, the distinctive histology of IMT-RAs dominated by epithilioid neoplastic cells also intrinsically reflects the heightened invasiveness of the tumor. However, it should be particularly noted that not all IMTs with round cell morphology carry the genetic alteration of IMT-RA [8]. Therefore, it is inappropriate to diagnosis IMT-RA based solely on morphologic features.

(3) The genetic features of the tumor: The fusion point of IMT-RAs reported to date constantly presents between exon 18 of *RANPB2* and exon 20 of *ALK* (Table 2). Sasaki [15] found that the *RANPB2-ALK* fusion gene could lead to interleukin (IL)-3 independent growth of Ba/F3 cells. Similarly, another study showed that bone marrow cells transfected with the *RANBP2-ALK* gene acquired an enhanced colony-forming potential and a decreased dependency on cytokine [16]. These studies suggested that the chimeric *RANPB2-ALK* gene could promote cellular proliferation, which might be a potential mechanism for the rapid regrowth and recurrence of IMT-RA. However, there is still a lack of direct experimental evidence linking the functions of this fusion gene with the increased aggressiveness of IMT-RA.

The article "Inflammatory myofibroblastic tumor with RANBP2 and ALK gene rearrangement: a report of two cases and literature review" was published in 2013. Journal: Diagn Pathol.

**Table 2:** **Genetic and immunohistochemical characteristics of 11 cases of inflammatory myofibroblastic tumor with *RANBP2-ALK *gene fusion**

**Case**	**Genetic features**		**Immunohistochemical features**							
	***RANBP2*to*ALK*fusion point**	**Detection techniques**	**ALK**	**Desmin**	**SMA**	**Caldesmin**	**CD30**	**CK**	**EMA**	**S100**
1	Exon 18 to exon 20	RT-PCR, FISH	NM+	/	/	/	/	/	/	/
2	Exon 18 to exon 20	RT-PCR, FISH	NM+	/	/	/	/	/	/	/
3	Exon 19 to exon 20^*^	RT-PCR, FISH	CP+	+	+	-	/	+	/	-
4	Exon 18 to exon 20	RT-PCR	NM+	-	-	/	-	-	/	-
5	Exon 18 to exon 20	RT-PCR	NM+	+	-	/	/	-	/	/
6	Exon 18 to exon 20	RT-PCR	NM+	+	-	-	+	-	-	-
7	Exon 18 to exon 20	RT-PCR	NM+	+	/	-	+	/	/	-
8	Exon 18 to exon 20	RT-PCR	NM+	+	+	-	+	-	/	-
9	Unknown	FISH	CP+	+	-	/	-	+	/	-
10	Unknown	FISH	NM+	+	+	-	+	-	-	-
11	Exon 18 to exon 20	RT-PCR, FISH	NM+	+	+	-	+	-	-	-
Total	/	/	100% (11/11)	89% (8/9)	50% (4/8)	0% (0/6)	71% (5/7)	25% (2/8)	0% (0/3)	0% (0/8)

*NM* nuclear membrane, *CP* cytoplasm.

^*^Reference 7 stated that the fusion point was exon 19 of *RANBP2* to exon 20 of *ALK*, while Figure 2 in the paper indicated that the actual fusion location was exon 18 of *RANBP2* to exon 20 of *ALK*.

From a diagnostic viewpoint, IMT-RA needs to be differentiated from a large group of tumors that manifest epithelioid features. Immunohistochemistry is greatly helpful in this process. Nuclear membrane staining of ALK is a unique immunophenotype of IMT-RA, which is observed in 82% (9/11) of cases. Unexplainably, a cytoplasmic pattern is also detected in 18% (2/11) of cases. In addition, the neoplasms display varied expression of desmin (89%, 8/9), CD30 (71%, 5/7), SMA (50%, 4/8), and cytokeratin (25%, 2/8), while EMA, S100, CD117, Myf4, myogenin, caldesmin, and HMB45 expression is consistently negative. Therefore, IMT-RAs could be easily distinguished from poorly differentiated carcinoma, malignant melanoma, epithelioid gastrointestinal stromal tumor, epithelioid solitary fibrous tumor [17], myofibroma [18] and alveolar rhabdomyosarcoma. It is noteworthy that a few mesenchymal mimics listed below may also show cytoplasmic ALK staining [19] and thus should particularly be discriminated to avoid misdiagnosis. (1) Epithelioid leiomyosarcoma (ELS): Compared with IMT-RA, ELS commonly displays greater cellular atypia and pleomorphism, and higher cellular density. ELS generally lacks an extensive myxoid background and inflammatory infiltrates. Furthermore, calponin and caldesmin expression could be recognized in ELS but not in IMT-RA [20]. (2) Inflammatory malignant fibrous histiocytoma (IMFH): Clinically, IMFH is more prone to occur in elderly individuals, which is different from IMT-RA that typically develops in young adults (median age, 34 years). Histologically, while the inflammatory infiltrates may be striking in both types of the tumors, the neoplastic cells in IMFH tend to be more pleomorphic, in contrast with the relative homogeneity in cellular morphology of IMT-RA. The neoplastic cells in IMFH are frequently fusiform and closely packed, and commonly arranged in a storiform pattern. Immunostaining of CD68 favors the diagnosis of IMFH. (3) Epithelioid malignant peripheral nerve sheath tumor (E-MPNST): Most E-MPNSTs develop from the setting of neurofibromatosis. E-MPNST presents with more or fewer spindled tumor cells in the lesion, and the myxoid stroma is more often focal rather than abundant [21,22]. Moreover, desmin and CD30 expression have not been discovered in E-MPNSTs. All of these features differ from those of IMT-RA. (4) Anaplastic large cell lymphoma (ALCL): The distinction between IMT-RA and ALCL has been described in a previous report [10]. Desmin and nuclear membrane ALK staining are suggestive of IMT-RA, as neither of these staining patterns has been observed in ALCL.

The article "Inflammatory myofibroblastic tumor with RANBP2 and ALK gene rearrangement: a report of two cases and literature review" was published in 2013. Journal: Diagn Pathol.

Most of the reported IMT-RAs are treated by surgical resection combined with chemotherapy. However, this therapeutic regimen seems to not effectively control the rapid recurrence of IMT-RAs. Recently, ALK inhibitor (ALKi) has been applied in the therapy of 2 IMT-RA cases, and a sustained partial response has been observed in at least 1 case [9]. Of note, the sensitivity of ALKi was reduced during standing treatment because of a secondary *ALK* gene mutation [15]. Thus, the long-term results of ALKi therapy remain to be further evaluated.

## Conclusions

In comparison with conventional IMTs, IMT-RAs show enhanced aggressive behaviors, which are possibly closely associated with their abdominopelvic origination, large tumor size, epithelioid tumoral morphology, and *RANPB2-ALK* gene rearrangement. An in-depth understanding on this entity is urgently needed to avoid misdiagnosis and provide effective treatment schedules.

## Consent

Written informed consents were obtained from the patient of Case 2 and the mother of the patient of Case 1 for publication of this report and accompanying images. The copies of the written consents are available for review by the Editor-in Chief of this Journal.

The article "Inflammatory myofibroblastic tumor with RANBP2 and ALK gene rearrangement: a report of two cases and literature review" was published in 2013. Journal: Diagn Pathol.

## Competing interests

The authors declare that they have no competing interests.

## Authors’ contributions

JL performed the histological, immunohistochemical and RT-PCR evaluation, literature review and drafted the manuscript. W-HY participated in histological diagnosis and immunohistochemical evaluation. KT performed FISH analysis and revised the manuscript. GH designed the study and literature review, and drafted the manuscript. Y-HH contributed to the literature review. JKCC participated in histological diagnosis and revised the manuscript. All authors read and approved the final manuscript.
